The article "Identification of Characteristic Genes in Whole Blood of Intervertebral Disc Degeneration Patients by Weighted Gene Coexpression Network Analysis (WGCNA)" was retracted in 2023. Reasons: signs of a paper mill; suspected computer-generated content; unreliable results or conclusions; concerns about the data.

# Identification of Characteristic Genes in Whole Blood of Intervertebral Disc Degeneration Patients by Weighted Gene Coexpression Network Analysis (WGCNA)

**DOI:** 10.1155/2022/6609901

**Published:** 2022-01-13

**Authors:** Xiaobo Ma, Junqiang Su, Bo Wang, Xiasheng Jin

**Affiliations:** Department of Orthopaedics, Yuncheng Central Hospital, Shanxi University, Yuncheng, China 044000

## Abstract

Intervertebral disc degeneration (IDD) is a major cause of lower back pain. However, to date, the molecular mechanism of the IDD remains unclear. Gene expression profiles and clinical traits were downloaded from the Gene Expression Omnibus (GEO) database. Firstly, weighted gene coexpression network analysis (WGCNA) was used to screen IDD-related genes. Moreover, least absolute shrinkage and selection operator (LASSO) logistic regression and support vector machine (SVM) algorithms were used to identify characteristic genes. Furthermore, we further investigated the immune landscape by the Cell-type Identification By Estimating Relative Subsets Of RNA Transcripts (CIBERSORT) algorithm and the correlations between key characteristic genes and infiltrating immune cells. Finally, a competing endogenous RNA (ceRNA) network was established to show the regulatory mechanisms of characteristic genes. A total of 2458 genes were identified by WGCNA, and 48 of them were disordered. After overlapping the genes obtained by LASSO and SVM-RFE algorithms, genes including LINC01347, ASAP1-IT1, lnc-SEPT7L-1, B3GNT8, CHRNB3, CLEC4F, LOC102724000, SERINC2, and LOC102723649 were identified as characteristic genes of IDD. Moreover, differential analysis further identified ASAP1-IT1 and SERINC2 as key characteristic genes. Furthermore, we found that the expression of both ASAP1-IT1 and SERINC2 was related to the proportions of T cells gamma delta and Neutrophils. Finally, a ceRNA network was established to show the regulatory mechanisms of ASAP1-IT1 and SERINC2. In conclusion, the present study identified ASAP1-IT1 and SERINC2 as the key characteristic genes of IDD through integrative bioinformatic analyses, which may contribute to the diagnosis and treatment of IDD.

## 1. Introduction

Intervertebral disc degeneration (IDD), a major cause of lower back pain and various degenerative spinal disorders, has been regarded as a global health issue because of the heavy burden on the healthcare system and severe economic consequences [1]. IDD can occur with the increasing of age, which is estimated to influence at least 5% of the population in developed countries each year [2, 3]. It was revealed that the apoptosis of nucleus pulposus (NP) cells and the degradation of the extracellular matrix are the main pathological changes that occur in IDD [4, 5]. The occurrence of IDD is affected by environmental and genetic factors, including aberrant gene expression, cell death, and inflammation [5–7]. Currently, although conservative and surgical treatment is considered the effective treatment to relieve pain of IDD patients, these treatments only can reduce the severity of symptoms but do not cure the disease [8, 9]. On the other hand, the diagnosis of IDD is difficult, which can greatly affect the treatment of IDD [10, 11]. Therefore, screening novel potential biomarkers for the diagnosis and treatment of IDD is needed.

The article "Identification of Characteristic Genes in Whole Blood of Intervertebral Disc Degeneration Patients by Weighted Gene Coexpression Network Analysis (WGCNA)" was retracted in 2023. Reasons: signs of a paper mill; suspected computer-generated content; unreliable results or conclusions; concerns about the data.

It is suggested that genetic change is the most dominant factor leading to the occurrence of IDD. For example, collagen type I alpha 1 chain (COL1A1) and collagen type I alpha 2 chain (COL1A2) can increase the risk of IDD by impairing the stability of collagens [12, 13]. Moreover, the genetic polymorphisms of parkin RBR E3 ubiquitin protein ligase (PARK2) and carbohydrate sulfotransferase 3 (CHST3) are associated with IDD occurrence [14, 15]. Furthermore, it was found that noncoding RNAs (ncRNAs, including microRNAs (miRNAs), long noncoding RNAs (lncRNAs), and circular RNAs (circRNAs)) also participate in the development of IDD by the competing endogenous RNA (ceRNA) network [16–19]. For instance, the inflammation-dependent downregulation of miR-194-5p can contribute to the pathogenesis of IDD through targeting cullin 4A (CUL4A) and cullin 4B (CUL4B) [16]. Furthermore, lncRNA HOTAIR can affect the IDD via the Wnt/*β*-catenin pathway [19]. lncRNA SNHG1 can promote NP cell proliferation by suppressing miR-326 expression and upregulating CCND1 expression [18]. circRNA VMA21 can alleviate inflammatory cytokine-induced NP cell apoptosis and imbalance between anabolism and catabolism of extracellular matrix through the miR-200c-XIAP pathway [17]. However, the molecular mechanisms of IDD remain unknown.

Increasing evidence has revealed that immune response plays an important role in the development of IDD [20–22]. It has been suggested that NP cells can activate the immune response once the blood-NP barrier is damaged, which is a crucial factor of IDD degeneration and can result in multiple pathological processes [20]. Moreover, studies have suggested that proinflammatory cytokines, such as interleukin-1*β* (IL-1*β*) and tumor necrosis factor-alpha (TNF-*α*), which are produced by immune cells, can induce degeneration and apoptosis of NP cells by activating *β*-catenin [21, 22]. Nevertheless, the immune landscape and regulatory mechanism of immune cells in IDD remain unclear.

In the present study, we firstly identified key characteristic genes related to IDD by the WGCNA using the gene expression profiles. Next, the immune landscape and the correlations between key characteristic genes and infiltrating immune cells were investigated. Finally, we further explored the regulatory mechanism of key characteristic genes. The integrated analysis of key characteristic genes and infiltrating immune cells would provide new biomarkers for the diagnosis and treatment of IDD.

The article "Identification of Characteristic Genes in Whole Blood of Intervertebral Disc Degeneration Patients by Weighted Gene Coexpression Network Analysis (WGCNA)" was retracted in 2023. Reasons: signs of a paper mill; suspected computer-generated content; unreliable results or conclusions; concerns about the data.

## 2. Materials and Methods

### 2.1. Data Acquisition

Three IDD-related gene expression profiles and clinical traits of the Chinese population, including GSE150408 and GSE124272, were downloaded from the Gene Expression Omnibus (GEO, https://www.ncbi.nlm.nih.gov/geo/) [23]. The GSE150408 dataset, including 17 whole blood samples of IDD patients and 17 whole blood samples of control samples, was used to construct a weighted gene coexpression network and identify differentially expressed genes (DEGs) between IDD and control samples. The GSE124272 dataset, including 8 whole blood samples of IDD patients and 8 whole blood samples of control samples, was selected as a validation set.

### 2.2. Construction of Weighted Gene Coexpression Network

We extracted the expression profile of IDD samples and control samples in the GSE150408 dataset to perform WGCNA by using the WGCNA package in R [24]. Firstly, we performed the sample cluster analysis by the hclust function to remove the outliers. Next, the pickSoftThreshold function was used to determine the soft thresholding power value to achieve an approximately scale-free network topology [25, 26]. Moreover, the adjacency matrix was transformed into a topological overlap matrix by quantitatively describing the similarity in nodes by comparing the weighted correlation between two nodes and other nodes. Furthermore, all genes were assigned into coexpression modules through a dynamic tree cutting algorithm by setting the minimal module size of 200 genes, and modules with highly correlated eigengenes (correlation above 0.3) were merged [27].

### 2.3. Identification of IDD-Related Module and Genes

To screen IDD-related modules, we calculated the correlation of clinical traits and the modules. The module with the highest correlation coefficient with IDD and *p* value < 0.05 was selected as IDD-related modules, and genes in the module were defined as IDD-related genes.

### 2.4. Identification of Differentially Expressed IDD-Related Genes

Firstly, differentially expressed genes (DEGs) between IDD samples and control samples were screened by limma package in R [28]. Genes with the threshold of *p* < 0.05 and ∣log_2_ Fold Change (FC) | >1.2 were defined as DEGs. Moreover, the volcano plot and heatmap of the DEGs were plotted by the ggplot2 package in R [29]. Finally, differentially expressed IDD-related genes were identified by overlapping the IDD-related genes and DEGs using the Venn diagram package in R [30], and we also plotted a heatmap to show the expression levels of the differentially expressed IDD-related genes through the pheatmap package in R [31].

The article "Identification of Characteristic Genes in Whole Blood of Intervertebral Disc Degeneration Patients by Weighted Gene Coexpression Network Analysis (WGCNA)" was retracted in 2023. Reasons: signs of a paper mill; suspected computer-generated content; unreliable results or conclusions; concerns about the data.

### 2.5. Gene Ontology (GO) and Kyoto Encyclopedia of Genes and Genomes (KEGG) Enrichment Analysis

To investigate the function of differentially expressed IDD-related genes, the KOBAS website (http://kobas.cbi.pku.edu.cn/) was used to perform the GO and KEGG enrichment analysis, and *p* < 0.05 were considered significant enrichment [32].

### 2.6. Identification and Validation of Characteristic Genes

To further identify characteristic genes from the differentially expressed IDD-related genes, least absolute shrinkage and selection operator (LASSO) logistic regression [33] and support vector machine (SVM) algorithms [34] were selected to perform feature selection to identify characteristic genes for IDD. The Glmnet package in R was used to implement LASSO analysis with the parameter setting as family =  ^“^binomial^”^ [35]. To avoid overfitting, 10-fold cross-validation was performed with the parameter setting as ^“^type.measure = auc.^”^ Moreover, the e1071 package in R was used to carry out SVM-RFE analysis through deleting SVM-generated eigenvectors [9]. To establish the SVM model based on Radial Basis Function and 10-fold cross-validation, the parameter was set as “*C* = 0.5 and gamma = 0.01.” Finally, genes overlapped in the LASSO algorithm and VM-RFE algorithm were selected as characteristic genes for further analysis. Furthermore, to screen the key characteristic genes, we further verify the expression levels of characteristic genes in the GSE124272 dataset.

### 2.7. Evaluation of Diagnostic Value of Key Characteristic Genes

To verify whether key characteristic genes can distinguish IDD samples and control samples in the GSE150408 and GSE124272 dataset, the receiver operating characteristic (ROC) curves were plotted to evaluate the diagnostic value of key characteristic genes by calculating the area under the ROC curves (AUCs) using the pROC package in R [36].

### 2.8. Correlation between Key Characteristic Genes and Infiltrating Immune Cells

To further investigate the correlation between key characteristic genes and infiltrating immune cells, we compared the proportion and composition of infiltrating immune cells in IDD samples and control samples in the GSE150408 dataset by the Cell-type Identification By Estimating Relative Subsets Of RNA Transcripts (CIBERSORT) algorithm based on a validated leukocyte gene signature matrix containing 547 genes and 22 human immune cell subpopulations [37]. Firstly, the gene expression matrix of the GSE150408 dataset was input in CIBERSORT for analysis based on a deconvolution algorithm with 100 permutations. Next, to make sure the accuracy of the deconvolution algorithm, samples with a CIBERSORT *p* > 0.05 were filtered out in the CIBERSORT analysis. In addition, the Wilcoxon rank-sum test was used to assess the differences in the proportion for infiltrating immune cells between UC samples and normal samples. Ultimately, a heatmap and a violin plot were plotted to show the difference of infiltrating immune cells between IDD samples and control samples by the pheatmap package in R and vioplot package in R [31], and the correlation heatmaps among infiltrating immune cells and between key characteristic genes and differentially infiltrating immune cells were drawn using the corrplot package in R [38].

The article "Identification of Characteristic Genes in Whole Blood of Intervertebral Disc Degeneration Patients by Weighted Gene Coexpression Network Analysis (WGCNA)" was retracted in 2023. Reasons: signs of a paper mill; suspected computer-generated content; unreliable results or conclusions; concerns about the data.

### 2.9. Construction of a ceRNA Network Based on the Key Characteristic Genes

To investigate the regulating regulatory mechanism of the key characteristic genes, we established a lncRNA-miRNA-mRNA network. Given that the key characteristic genes might include protein-coding genes and noncoding genes, we firstly predicted the target miRNAs of key characteristic lncRNAs in the LncBase database. Next, we predicted the target genes of miRNAs in the miRDB, TargetScan, and miRTarBase and acquired the overlapping target genes. Finally, intersection genes of overlapping target genes and DEGs were obtained and used to construct a ceRNA network. Similarly, we firstly predicted the regulating miRNAs of key characteristic protein-coding genes in the miRWalk and miRDB database and obtained overlapping miRNAs. Moreover, the regulating lncRNAs of overlapping miRNAs were predicted by the starbase database. Furthermore, intersection genes of regulating lncRNAs and DEGs were used to construct a ceRNA network. Ultimately, Cytoscape v 3.7.1 was used to present the ceRNA network.

### 2.10. Statistical Analysis

All statistical analyses were performed by R Studio (R Version 4.0.2) software. The Wilcoxon rank-sum test was used to compare the difference between two different groups. *p* value < 0.05 was set as the standard of statistical analysis. The results were expressed as the median with interquartile range.

## 3. Results

### 3.1. Identification of IDD-Related Module and Genes

To identify genes related to IDD, a weighted coexpression network was constructed. Sample clustering suggested that 4 samples were outliers and were filtered out in the subsequent analysis (Figure 1(a)). A total of 22 modules were identified by setting the soft threshold power of *β* (scale-free R2 = 0.94) as 14, which could satisfy the distribution of a scale-free network (Figure 1(b)), and merging modules whose eigengenes were correlated above 0.3 (Figure 1(c)). Moreover, the analysis of the relationship of the modules and the traits revealed that the brown module was significantly positively correlated with IDD (Figure 1(d), *p* < 0.05, and correlation coefficient = 0.39). Therefore, the brown module was defined as the IDD-related module, and 2458 genes in this module were defined as IDD-related genes.

The article "Identification of Characteristic Genes in Whole Blood of Intervertebral Disc Degeneration Patients by Weighted Gene Coexpression Network Analysis (WGCNA)" was retracted in 2023. Reasons: signs of a paper mill; suspected computer-generated content; unreliable results or conclusions; concerns about the data.

### 3.2. Identification of Differentially Expressed IDD-Related Genes

Under the criteria of ∣log_2_ (FC) | >1.2 and *p* value < 0.05, a total of 253 genes, including 134 upregulated genes and 119 downregulated genes, were identified as DEGs between IDD samples and control samples in the GSE150408 dataset (Figure 2(a)). After overlapping IDD-related genes and DEGs, 48 genes were selected as differentially expressed IDD-related genes for further analyses (Figure 2(b)). Moreover, as shown in Figure 2(c), most of the differentially expressed IDD-related genes were upregulated in TDD samples compared to control samples.

### 3.3. GO and KEGG Enrichment Analysis

To explore the biological function of differentially expressed IDD-related genes, we performed the GO and KEGG enrichment analysis by the KOBAS website. The result of GO analysis suggested that these genes were mainly associated with carbohydrate binding, skeletal system development, transmembrane signaling receptor activity, tertiary granule lumen, and human leukocyte antigens (HLA) in humans (MHC) class I receptor activity-related biological processes (Figure 3(a)). Moreover, for KEGG pathway analysis, these genes were mainly involved in relaxin signaling pathway, proximal tubule bicarbonate reclamation, and so on (Figure 3(b)). Therefore, these genes might play a key role in IDD by regulating these biological processes and signaling pathways.

### 3.4. Identification and Validation of Characteristic Genes

The LASSO algorithm and SVM-RFE algorithm were selected to identify characteristic genes from the 48 differentially expressed IDD-related genes. Firstly, the LASSO logistic regression algorithm identified 9 characteristic genes, including LINC01347, ASAP1-IT1, lnc-SEPT7L-1, B3GNT8, CHRNB3, CLEC4F, LOC102724000, SERINC2, and LOC102723649, as characteristic genes (Figures 4(a) and 4(b)). Moreover, 22 genes, including lnc-SEPT7L-1, CA4, CLEC4F, LINC01347, B3GNT8, SERINC2, lnc-ZNF37A-3, ASAP1-IT1, CRISPLD2, C18orf32, LOC102724000, SHOX2, lnc-CLGN-2, LOC729737, LOC101926894, LOC441124, LOC102724552, LOC102723649, CHRNB3, lnc-HNRNPA3-1, ZNF107, and LOC101926936, were screened as characteristic genes using the SVM-RFE algorithm (Figures 4(c) and 4(d)). Finally, LINC01347, ASAP1-IT1, lnc-SEPT7L-1, B3GNT8, CHRNB3, CLEC4F, LOC102724000, SERINC2, and LOC102723649 were identified as characteristic genes by overlapping the genes obtained by the two algorithms (Figure 4(c)). In order to further verify the expression levels of these 9 characteristic genes, we further conducted the differential expression analysis in the GSE124272 dataset and found that the expression of ASAP1-IT1 and SERINC2 were markedly different between IDD and control samples (*p* value < 0.05). As shown in Figure 5(a), the expression of both ASAP1-IT1 and SERINC2 was upregulated in IDD samples compared to control samples. Interestingly, both ASAP1-IT1 and SERINC2 showed higher expression in IDD samples compared to control samples in the GSE150408 dataset (Figure 5(b)). Thus, these two genes were selected as key characteristic genes.

The article "Identification of Characteristic Genes in Whole Blood of Intervertebral Disc Degeneration Patients by Weighted Gene Coexpression Network Analysis (WGCNA)" was retracted in 2023. Reasons: signs of a paper mill; suspected computer-generated content; unreliable results or conclusions; concerns about the data.

### 3.5. Evaluation of Diagnostic Value of Key Characteristic Genes

To verify whether key characteristic genes can distinguish IDD samples and control samples, the ROC curves were plotted to evaluate the diagnostic value of key characteristic genes by calculating the AUC values. Pleasingly, ROC analyses revealed that both the AUCs of ASAP1-IT1 and SERINC2 for distinguishing IDD samples and control samples were greater than 0.7 in the GSE150408 and GSE124272 datasets (Figures 6(a) and 6(b)), which indicated that ASAP1-IT1 and SERINC2 could be used as the diagnostic biomarkers.

### 3.6. Correlation between Key Characteristic Genes and Infiltrating Immune Cells

To further investigate the correlation between key characteristic genes and infiltrating immune cells, we compared the proportion and composition of infiltrating immune cells in IDD samples and control samples in the GSE150408 dataset by the CIBERSORT algorithm. As shown in Figures 7(a) and 7(b), the proportions of plasma cells, T cells gamma delta, and Neutrophils presented a significant difference between IDD samples and control samples. Moreover, the correlation analysis of infiltrating immune cells revealed that the proportions of T cells gamma delta and Neutrophils had a negative correlation (Figure 7(c)). Interestingly, the correlation analysis between key characteristic genes and differently infiltrating immune cells suggested that the expression of both ASAP1-IT1 and SERINC2 was negatively related to the proportions of T cells gamma delta (Figure 7(d)). Moreover, the expression of SERINC2 was positively related to the proportions of Neutrophils (Figure 7(d)). Therefore, ASAP1-IT1 and SERINC2 might be associated with the immune response in IDD by regulating the proportions of T cells gamma delta and Neutrophils.

The article "Identification of Characteristic Genes in Whole Blood of Intervertebral Disc Degeneration Patients by Weighted Gene Coexpression Network Analysis (WGCNA)" was retracted in 2023. Reasons: signs of a paper mill; suspected computer-generated content; unreliable results or conclusions; concerns about the data.

### 3.7. Construction of a ceRNA Network Based on the Key Characteristic Genes

To further explore the regulatory mechanisms of ASAP1-IT1 and SERINC2, we constructed a ceRNA network. Notably, ASAP1-IT1 is a lncRNA, but SERINC2 is a protein-coding gene. Thus, we firstly predicted target 168 miRNAs and 3780 protein-coding genes of ASAP1-IT1. Moreover, 5 regulating miRNAs and 168 lncRNAs of ASAP1-IT1 were predicted. Finally, a ceRNA network, including 12 protein-coding genes, 172 miRNAs, and 1 lncRNAs, was constructed. As shown in Figure 8, ASAP1-IT1 might regulate ACAD8, GK5, CRISPLD2, ZBTB37, TMEM64, ARL5B, FNBP1L, CD86, SHOX2, ZNF107, TBPAN13, and SERINC2. Therefore, we speculated that ASAP1-IT1 might affect the immune response in IDD by regulating SERINC2.

## 4. Discussion

IDD, a multifactorial disease, has become a major contributor to radicular back and neck pain. The mechanism of the occurrence of IDD is complex and influenced by various factors, such as mechanical stress, aging, inflammation, and infection [22, 39, 40]. Currently, existing treatments do not cure IDD or reverse the progression of IDD, insufficiently. Moreover, the early diagnosis of IDD is difficult. The less effective diagnosis and treatment of IDD seriously affect the life of IDD patients and bring a heavy economic burden to society [41]. Luckily, gene expression profiles provide the convenience for screening novel biomarkers in neoplastic and nonneoplastic diseases [42, 43]. Therefore, we aimed to identify characteristic genes for IDD and further investigate the correlations of immune cells and characteristic genes.

Firstly, we obtained the IDD expression profiles from the GEO database. Next, WGCNA identified 2458 IDD-related genes, and 48 of them were disordered. GO and KEGG enrichment analysis suggested that these differentially expressed IDD-related genes were mainly involved in MHC class I receptor activity and relaxin signaling pathway. It has been revealed that MHC class I receptor activity is associated with immune response [44]. The relaxin pathway is related to osteoblast differentiation and bone formation [45]. Therefore, we speculated that these 48 differentially expressed IDD-related genes might play key roles in IDD by regulating immune response, osteoblast differentiation, and bone formation. Moreover, LINC01347, ASAP1-IT1, lnc-SEPT7L-1, B3GNT8, CHRNB3, CLEC4F, LOC102724000, SERINC2, and LOC102723649 were identified as characteristic genes by overlapping the genes obtained by the LASSO and SVM-RFE algorithm. Finally, ASAP1-IT1 and SERINC2 were selected as the key characteristic genes by the differential analysis and showed well diagnostic significance. To our knowledge, there is no report about the role of ASAP1-IT1 in IDD. In our study, we firstly found that ASAP1-IT1 might affect the occurrence or development of IDD and be used to diagnose IDD. However, it has been suggested that ASAP1-IT1 can influence the progression by regulating the hedgehog signaling pathway [46]. Moreover, upregulation of ASAP1-IT1 can affect the metastasis of non-small-cell lung cancer by introducing the PTEN/AKT signaling pathway [47]. Furthermore, ASAP1-IT1 has been proven to be a tumor suppressor lncRNA in ovarian cancer by mediating the Hippo/YAP signaling pathway [48]. Thus, we speculated that ASAP1-IT1 may play an important role in IDD. Similarly, there is no report about the role of SERINC2 in IDD. However, recent research found that suppressing the expression of SERINC2 is related to the progression of lung adenocarcinoma by influencing the PI3K/AKT signaling pathway [49]. SERINC2 have been reported to affect the prognosis of low-grade glioma [50]. Nevertheless, further study about the role of ASAP1-IT1 and SERINC2 in IDD is needed.

The article "Identification of Characteristic Genes in Whole Blood of Intervertebral Disc Degeneration Patients by Weighted Gene Coexpression Network Analysis (WGCNA)" was retracted in 2023. Reasons: signs of a paper mill; suspected computer-generated content; unreliable results or conclusions; concerns about the data.

Given the significance of immune response in IDD, we further compared the proportions of immune cells between IDD samples and control samples and found that the proportions of plasma cells, T cells gamma delta, and Neutrophils were significantly different in IDD samples and control samples. In particular, the proportion of Neutrophils was significantly higher in IDD samples compared to control samples, but the proportion of T cells gamma delta was significantly lower in IDD samples compared to control samples. Plasma cells, which are derived from B cells, are the only cell type in the organism that can produce antibodies. It has been suggested that plasma cells are related to the production of different cytokines, such as IL-10, IL-35, IL-17, GM-CSF, and iNOS [51–53]. Notably, IL-37 is a new member of the IL-1 family that plays a key role in the IDD by acting as a master regulator [54]. T cells gamma delta is a subset of T lymphocytes that comprise 5% of the peripheral lymphocyte population. Researches have suggested that T cells gamma delta can recognize nonprotein phosphoantigens, isoprenoid pyrophosphates, alkylamines, nonclassic MHC class I molecules, MICA, and MICB molecules, as well as hsp-derived peptides without requiring antigen processing and MHC presentation [55–57]. Moreover, T cells gamma delta also can present the Th1-, Th2-, Th17-, and Treg-like phenotype and function as a regulator for the inflammation [58]. Furthermore, T cells gamma delta has been revealed to play an important role in the regulation of various autoimmune diseases [59, 60, 66]. Neutrophils, also known as polymorphonuclear leukocytes, are mainly associated with host defense [61]. Neutrophils can deliver a signal to other immune cells by secreting cytokines and chemokines [62, 63]. On the other hand, the imbalance of Neutrophils can aggravate the disease. For example, the occurrence of rheumatoid arthritis can recruit Neutrophils and lead to tissue damage and ultimately result in irreversible processes like cartilage destruction [64]. Therefore, plasma cells, T cells gamma delta, and Neutrophils may play a critical role in IDD through regulating immune and inflammatory responses. Interestingly, ASAP1-IT1 was negatively correlated with T cells gamma delta and SERINC2 was related to the proportions of T cells gamma delta and Neutrophils. Thus, we speculated that ASAP1-IT1 and SERINC2 may also affect the IDD by regulating T cells gamma delta and Neutrophils.

The article "Identification of Characteristic Genes in Whole Blood of Intervertebral Disc Degeneration Patients by Weighted Gene Coexpression Network Analysis (WGCNA)" was retracted in 2023. Reasons: signs of a paper mill; suspected computer-generated content; unreliable results or conclusions; concerns about the data.

Interestingly, the ceRNA network showed that ASAP1-IT1 might regulate SERINC2. Thus, ASAP1-IT1 might play a key role in immune response of IDD by regulating SERINC2. However, further verification of regulating relationships is necessary.

## 5. Conclusion

In conclusion, we identified ASAP1-IT1 and SERINC2 as the key characteristic genes of IDD through integrative bioinformatic analyses. Moreover, we also that found the expression of ASAP1-IT1 and SERINC2 was associated with the proportions of T cells gamma delta and Neutrophils. Finally, we also found that ASAP1-IT1 might regulate SERINC2. In short, ASAP1-IT1 and SERINC2 might be used as biomarkers for the diagnosis and treatment of IDD. However, further researches are urgent to verify the roles of ASAP1-IT1 and SERINC2 in IDD and the regulatory mechanism.

## Figures and Tables

**Figure 1:** Construction of weighted gene coexpression network and identification of module related to IDD. (a) Sample cluster analysis identified the outlier samples in the GSE150408 dataset. (b) Determination of the optimal soft threshold to conform to the scale-free distribution. (c) Dendrogram of genes clustered based on the highly correlated eigengenes (correlation above 0.3). (d) Heatmap of the correlation between module eigengenes and clinical traits.

**Figure 2:** Identification of differentially expressed IDD-related genes. (a) Volcano plot of the DEGs between IDD samples and control samples. (b) Overlapping genes between DEGs and genes in brown module. (c) Heatmap exhibited the expression levels of the differentially expressed IDD-related genes between IDD samples and control samples.

**Figure 3:** GO KEGG pathway enrichment analysis for the differentially expressed IDD-related genes. (a) GO terms enriched by the differentially expressed IDD-related genes. (b) KEGG pathways enriched by the differentially expressed IDD-related genes.

The article "Identification of Characteristic Genes in Whole Blood of Intervertebral Disc Degeneration Patients by Weighted Gene Coexpression Network Analysis (WGCNA)" was retracted in 2023. Reasons: signs of a paper mill; suspected computer-generated content; unreliable results or conclusions; concerns about the data.

**Figure 4:** Identification of characteristic genes for IDD. (a) log (Lambda) value of the differentially expressed IDD-related genes in the LASSO model. (b) The most proper log (Lambda) value in the LASSO model. (c, d) Support vector machine-recursive feature elimination algorithm to screen characteristic genes. (e) Venn diagram showed the overlapped genes obtained by the LASSO algorithm and VM-RFE algorithm.

**Figure 5:** The expression levels of characteristic genes. (a) The expression levels of characteristic genes in the GSE124272 dataset. (b) The expression levels of characteristic genes in the GSE150408 dataset.

**Figure 6:** Evaluation of diagnostic value of key characteristic genes. (a) ROC curves for key characteristic genes in the GSE124272 dataset. (b) ROC curves for key characteristic genes in the GSE150408 dataset.

**Figure 7:** Correlation between key characteristic genes and infiltrating immune cells. (a) Heatmap for the differences of infiltrating immune cells between IDD samples and control samples. (b) Violin plot showed the differences of infiltrating immune cells between IDD samples and control samples. (c) Correlation among infiltrating immune cells. (d) Correlation among key characteristic genes and differentially infiltrating immune cells.

**Figure 8:** The ceRNA network based on the key characteristic genes.

## Data Availability

The datasets (GSE150408 and GSE124272) included in the present study can be found in the GEO database (https://www.ncbi.nlm.nih.gov/geo/).
